# Clinical Efficacy of Modified *Yiwei Shengyang* Decoction Combined with FOLFOX4 Chemotherapy Regimen in the Treatment of Advanced Gastric Cancer and Its Effect on Tumor Marker Levels

**DOI:** 10.1155/2022/6234032

**Published:** 2022-05-05

**Authors:** Hongying Wu, Xiaomei Miao, Yan Liu, Shu Zhang, Chaohui Li, Jie Hao

**Affiliations:** ^1^National Physician Hall, Cangzhou Central Hospital, Cangzhou, China; ^2^Department of Hepatopancreatobiliary Surgery, Cangzhou Central Hospital, Cangzhou, China; ^3^Department of Oncology, Cangzhou Central Hospital, Cangzhou, China

## Abstract

**Objective:**

To study the clinical efficacy of modified *Yiwei Shengyang* decoction combined with FOLFOX4 chemotherapy regimen in the treatment of advanced gastric cancer and its effect on tumor marker levels.

**Methods:**

A total of 106 patients with advanced gastric cancer who were treated in our hospital from September 2019 to September 2021 were recruited and assigned via random number allocation to receive either FOLFOX4 chemotherapy (control group) or modified *Yiwei Shengyang* decoction plus FOLFOX4 chemotherapy (observation group). Outcome measures included clinical efficacy and tumor marker levels.

**Results:**

Modified *Yiwei Shengyang* decoction plus FOLFOX4 chemotherapy was associated with a significantly higher efficacy (86.79%, including 22 (41.51%) cases of complete response (CR), 24 (45.28%) cases of partial response (PR), 6 (11.32%) cases of stable disease (SD), and 1 (1.89%) case of progressive disease (PD)) compared to FOLFOX4 chemotherapy alone (47.16%, including 10 (18.87%) cases of CR, 15 (28.30%) cases of PR, 21 (39.62%) cases of SD, and 7 (13.21%) cases of PD) (*P* < 0.05). There was no significant difference in the levels of CEA and CA19-9 between the two groups before treatment (*P* > 0.05). Modified *Yiwei Shengyang* decoction plus FOLFOX4 chemotherapy resulted in significantly lower levels of carcinoembryonic antigen (CEA) and carbohydrate antigen 19-9 (CA19-9) (2.08 ± 0.47, 15.12 ± 6.74) compared to FOLFOX4 chemotherapy alone (5.46 ± 1.84, 31.82 ± 7.48) (*P* < 0.05).

**Conclusion:**

Modified *Yiwei Shengyang* decoction plus FOLFOX4 chemotherapy regimen is effective in the treatment of advanced gastric cancer. It regulates the levels of various serum tumor markers in patients and controls the disease, so it is worthy of clinical application and promotion.

## 1. Introduction

Gastric carcinoma [1], a malignant tumor originating from the gastric mucosa epithelium, is one of the common tumors of the digestive tract and ranks first in the incidence of various malignant tumors in China. The contributors to the high incidence and mortality of gastric cancer include local recurrence and distant metastasis [2]. Epidemiological statistics reveal that aggravation of environmental pollution and changes in dietary structure are the contributing factors to the increasingly rising prevalence of the disease. The 5-year survival rate of radical resection for early gastric cancer can reach 90%, while that of advanced gastric cancer is only 30%–40%. However, due to the atypical symptoms of gastric cancer in the early stage, most patients have progressed to an advanced stage by the time of diagnosis [3, 4]. Reportedly, 80%–90% of advanced gastric cancer patients are considered inoperable or experience recurrence within 5 years after surgery. As such, the unsatisfactory surgical treatment prompts targeted systemic chemotherapy [5, 6], among which the first-line chemotherapy drugs mainly include fluorouracils, taxanes, clamps, anthracyclines, and topoisomerase inhibitors. The FOLFOX4 regimen (oxaliplatin + 5-fluorouracil) [7] is the first choice for patients with gastric cancer, but it is prone to collateral damage to normal human cells, which may result in low compliance of patients and thus a shortened survival [8, 9]. Oxaliplatin is one of the single agents commonly used in the treatment of advanced gastrointestinal tumors. Its main pharmacological mechanism is to interfere with the normal replication and transcription of DNA by covalently binding to G on the DNA strand, producing intrastrand crosslinks and DNA crosslinks that result in DNA damage through the formation of complexes. The drug can also produce cytotoxicity and induce tumor cell death. Relevant studies have shown that chemotherapy might be associated with many adverse reactions, such as gastrointestinal reactions, bone marrow suppression, and other complications, resulting in poor tolerance and overall efficacy [10].

Traditional Chinese medicine believes that chemotherapy drugs can be detrimental to the lung *qi* and healthy *qi*, resulting in a deficiency of *qi* and blood and aggravating the dysfunction of the spleen. Modified *Yiwei Shengyang* decoction contains *Hedyotis diffusa*, *Astragalus*, *Poria*, wine-made peony, *Atractylodes*, ginseng, *Pinellia*, liquiritiae radix, Bupleurum, orange peel, *Alisma*, *Scutellaria barbata*, leech, and goldthread root and can exert the function of invigorating the spleen and benefiting the lung, soothing the liver and relieving stagnation, expelling wind and dampness, promoting blood circulation and removing blood stasis, and removing dampness and heat. In recent years, traditional Chinese medicine has achieved remarkable results in the treatment of advanced gastric cancer, with effective disease control and a reduced incidence of adverse reactions during chemotherapy [11]. Traditional Chinese medicine believes that chemotherapy drugs can damage lung qi, resulting in a deficiency of qi and blood and aggravating the deficiency of spleen and stomach, so the treatment principle is to benefit the stomach, strengthen the spleen and raise the yang. Traditional Chinese medicine combined with chemotherapy can significantly improve the quality of life of gastric cancer patients and enhance their immune function [5, 6]. Therefore, this paper aims to study and analyze the clinical efficacy of modified *Yiwei Shengyang* decoction combined with FOLFOX4 chemotherapy in the treatment of advanced gastric cancer and its effect on the level of tumor markers, aiming to provide an alternative for the clinical treatment of advanced gastric cancer.

## 2. Materials and Methods

### 2.1. Study Population

A total of 106 patients with advanced gastric cancer who were treated in our hospital from September 2019 to September 2021 were randomized at 1 : 1 ratio either to the observation group or control group via the random number method. The baseline data of the observation group (30 males and 23 females; aged 39–63 years, with an average age of 50.11 ± 5.13 years; 32 cases of adenocarcinoma, 12 cases of mucinous adenocarcinoma, and 9 cases of signet ring cell carcinoma) were comparable with those of the control group (27 males and 26 females; aged 37–60 years, with an average age of 49.98 ± 5.34 years; 34 cases of adenocarcinoma, 11 cases of mucinous adenocarcinoma, and 8 cases of signet ring cell carcinoma) (*P* > 0.05) (Table 1). The studies involving human participants were reviewed and approved by the Cangzhou Central Hospital, no. CCH29717.

### 2.2. Inclusion and Exclusion Criteria

Inclusion criteria: ① all met the diagnostic criteria for gastric cancer formulated by the American Joint Committee on Cancer (AJCC), and TNM stage was IIIB or above; ② patients with traditional Chinese medicine syndromes conforming to the *Guiding Principles of Clinical Research on New Chinese Medicines* for spleen-stomach weakness syndrome and epigastric distention or dull pain, fatigue, loose stools, sallow complexion, pale tongue, and thin and weak pulse; ③ no other malignant tumors.

Exclusion criteria: ① allergies to related drugs; ② dysfunction of vital organs such as heart, liver, and kidney; ③ complicated with coagulation disorders.

### 2.3. Research Methods

The control group was given FOLFOX4 chemotherapy regimen [12]: oxaliplatin injection (batch number HIE09099003, Qilu Pharmaceutical Co., Ltd.) 85 mg/m^2^ was given intravenously for 2 hours on day 1, 2 h intravenous drip of leucovorin injection (batch number 1002923, Jiangsu Hengrui Pharmaceutical Co., Ltd.) 200 mg/m^2^, intravenous bolus injection of 5-fluorouracil (batch number 090709, Shanghai Xu Donghaipu Pharmaceutical Co., Ltd.) 400 mg/m^2^, followed by continuous 2 h intravenous 5-fluorouracil 600 mg/m^2^ on days 1 and 2. One course of treatment was repeated every 2 weeks, with a total of 4 courses of treatment.

The patients in the observation group were treated with modified *Yiwei Shengyang* decoction plus FOLFOX4 chemotherapy (same as the control group). The components of the modified *Yiwei Shengyang* decoction include *Astragalus*, *Codonopsis* 30 g, *Poria* 20 g, 15 g each of white peony root, bark lotus, *Hedyotis diffusa*, and *Atractylodes*, 10 g each of tangerine peel, *Saposhnicovia divaricata*, *Pinellia*, *Alisma*, and 5 g licorice, decocted with water, 1 dose/d and taken 0.5 h after breakfast and dinner. A course spans 14 days, and 3 courses of treatment were given. The patients were routinely treated with antiallergy, hydration diuresis and antiemetic symptomatic treatment according to the daily observation.

### 2.4. Observation Indicators

① Clinical efficacy: according to the New Response Evaluation Criteria in Solid Tumors (RECIST) developed by the World Health Organization (WHO), the effectiveness is classified into complete response (CR), partial response (PR), stable disease (SD), and progressive disease (PD). CR: the target lesion completely disappeared after treatment and was maintained for at least 1 month. PR: the target lesion was significantly improved after treatment, and the sum of its maximum diameters decreased by ≥30%. The improvement was maintained for at least 1 month. SD: the target lesion had improved, but the reduction or increase of the sum of the maximum diameters was beyond the range of PR and PD. PD: after 3 cycles of treatment, the sum of the maximum diameters of target lesions increased by ≥20% compared with that before treatment, or new lesions appeared. Total efficacy = (CR cases + PR cases)/total number of cases *×* 100%.

② Tumor markers: 2–5 ml of fasting venous blood was collected from all patients and placed in a drying tube to prepare serum samples. The electrochemiluminescence immunoassay (ECLIA) was used to determine serum levels of the highly specific gastrointestinal tumor-associated antigen CA19-9 (Abcam, ab289665) and carcinoembryonic antigen (CEA, Abcam, ab133633) using automatic chemiluminescence immunoassay and original supporting reagents.

### 2.5. Statistical Analysis

SPSS22.0 software was used to process the data, and the enumeration data (*n* (%)) and measurement data ($\bar{x}$ ± *s*) were subjected to chi-square test and *t*-test, respectively. Differences were considered statistically significant at *P* < 0.05.

## 3. Results

### 3.1. Clinical Efficacy

Modified *Yiwei Shengyang* decoction plus FOLFOX4 chemotherapy was associated with a significantly higher efficacy (86.79%, including 22 (41.51%) cases of complete response (CR), 24 (45.28%) cases of partial response (PR), 6 (11.32%) cases of stable disease (SD), and 1 (1.89%) case of progressive disease (PD)) compared to FOLFOX4 chemotherapy alone (47.16%, including 10 (18.87%) cases of CR, 15 (28.30%) cases of PR, 21 (39.62%) cases of SD, and 7 (13.21%) cases of PD) (*P* < 0.05) (Table 2).

### 3.2. Tumor Markers

There was no significant difference in the levels of CEA and CA19-9 between the two groups before treatment (*P* > 0.05). Modified *Yiwei Shengyang* decoction plus FOLFOX4 chemotherapy resulted in significantly lower levels of CEA and CA19-9 (2.08 ± 0.47, 15.12 ± 6.74) versus FOLFOX4 chemotherapy alone (5.46 ± 1.84, 31.82 ± 7.48) (*P* < 0.05) (Table 3).

## 4. Discussion

According to statistics, the new cases and deaths of gastric cancer in China in 2015 accounted for 42.6% and 45.0% of the global total, respectively. As previously noted, effective control of cancer cell metastasis is the key to the treatment of advanced gastric cancer. The FOLFOX4 chemotherapy regimen can achieve effective disease control with a well-recognized efficacy [13]. However, due to its low selectivity to tumor cells and the poor adherence, the overall effect has been moderated [14].

According to traditional Chinese medicine, gastric cancer is categorized as “epigastric pain,” “accumulation of symptoms,” and “stomach accumulation.” The disease is located in the stomach, and the deficiency of healthy *qi* is the fundamental cause. The obstruction of the blood and blood vessels will lead to the loss of the healthy *qi*, and insufficient healthy *qi* will result in the imbalance of *yin* and *yang*. Moreover, long-term dietary disorders, weakness of the spleen and stomach, dysfunction of the internal organs, and the internal growth of evil toxins and eventually lead to blood stasis [15, 16]. Chemotherapy is detrimental to the healthy *qi* and causes deficiency of the spleen. The spleen and stomach are the foundation of acquired and the source of *qi* and blood. As a result, chemotherapy is associated with imbalanced *yin* and *yang* and declined organ function [17]. Therefore, the treatment focuses on raising *yang*, eliminating dampness, and strengthening the spleen.

In this study, given the deficiency of spleen qi and the dysfunction of upgrading the positive qi and lowering the evil qi after chemotherapy, the treatment centered on promoting yang and benefiting the stomach, strengthening the spleen, and drying dampness. Modified *Yiwei Shengyang* decoction was originally prepared by Li Dongyuan [11]. In the prescription, *Astragalus* is used as the monarch medicine, *Alisma*, *Poria*, *Pinellia*, *Atractylodes*, and *Codonopsis* are the minister medicines, and *Saposhnicovia divaricata*, *Paeonia lactiflora*, *Hedyotis diffusa*, etc., are used as adjuvants. *Astragalus* has the functions of invigorating *qi* and solidifying the exterior, diuretic, and expelling toxins, expelling pus, astringing sores, and promoting muscle. *Poria* is beneficial to the heart and can soothe the mind. *Atractylodes* can dissolve turbidity and relieve pain. Ginseng can nourish the five internal organs, soothe the spirit, calm the soul, relieve palpitation, eliminate unhealthy *qi*, and benefit intellectuality. *Pinellia* dries dampness, resolves phlegm, reduces inversion, relieves vomiting, and mitigates swelling. *Atractylodes* rhizoma has the functions of invigorating the spleen and nourishing *qi,* drying dampness and diuretic water, antiperspirant, tocolysis, and releasing heat [18].

Modern pharmacology has confirmed that *Saposhnicovia divaricata* and *Hedyotis diffusa* have remarkable antitumor effects. A combination of various medicines can nourish *qi* and strengthen the spleen, eliminate dampness, strengthen the body, and remove pathogenic factors, to achieve sufficient healthy *qi* and balance of yin and *yang* [19]. With the continuous development of immunology and molecular biology, tumor markers are playing an increasingly significant role in tumor screening, early diagnosis, prognosis prediction, and outcome evaluation. Tumor markers are a class of specific indicators that reflect the presence and growth of tumors, with a certain value in the auxiliary diagnosis, differential diagnosis, and curative effect observation of tumors. Therefore, the present study aimed to study and analyze modified *Yiwei Shengyang* decoction combined with FOLFOX4 chemotherapy regimen in the treatment of advanced gastric cancer and its effect on tumor marker levels.

The results of the present study showed that modified *Yiwei Shengyang* decoction plus FOLFOX4 chemotherapy was associated with a significantly higher efficacy versus FOLFOX4 chemotherapy alone, indicating that modified *Yiwei Shengyang* decoction combined with FOLFOX4 chemotherapy regimen yields an enhanced treatment efficacy and better disease control versus monotherapy of FOLFOX4 regimen. The possible explanation is that the gastrointestinal reactions and myelosuppression complications after chemotherapy result in more nutritional dysfunction and then disease aggravation. Modified *Yiwei Shengyang* decoction contains herbal medicines such as *Astragalus*, *Codonopsis*, and *Pinellia*, which nourish stomach-*yin* and can regulate the function of the gastrointestinal tract, thereby improving the nutritional function and facilitating the recovery of patients. The compatibility of the drugs in modified *Yiwei Shengyang* decoction focuses on drying dampness and stomach, strengthening the body, and eliminating pathogenic factors, which can effectively prevent the occurrence of adverse reactions such as nausea, hemoglobin decline, and gastrointestinal reactions, and help reduce adverse reactions. Both CEA and CA19-9 are common clinical serum tumor markers of gastric cancer. CEA and CA19-9 are common clinical serum tumor markers for gastric cancer. CEA is expressed in various malignant tumor tissues, and its expression is positively correlated with the severity of tumor development, with a sensitivity of about 30 W in gastric cancer patients. CA19-9 is a highly specific GI tumor-associated antigen whose expression is positively correlated with the degree of tumor development and is an important indicator of gastric cancer independently of other gastric cancer risk factors. To date, a large body of evidence has confirmed the important clinical significance of serum CEA and CA19-9 in the diagnosis and treatment of gastric cancer. The results of the present study showed that modified *Yiwei Shengyang* decoction plus FOLFOX4 chemotherapy resulted in significantly lower levels of CEA and CA19-9 versus FOLFOX4 chemotherapy alone, which is consistent with the results of previous studies. The limitations of this study lie in the absence of adverse drug reaction detection and long-term follow-up investigation. Long-term follow-up trials will be conducted in the future to obtain more reliable clinical data.

## 5. Conclusion

Modified *Yiwei Shengyang* decoction combined with FOLFOX4 chemotherapy regimen is effective in the treatment of advanced gastric cancer. It regulates the levels of various serum tumor markers in patients and controls the disease, so it is worthy of clinical application and promotion.

## Figures and Tables

**Table 1:** Baseline data ($\bar{x}$ ± *s*).

Groups	*N*	Gender		Age		Pathological type		
		Male	Female	Range	Mean age	Adenocarcinoma	Mucinous adenocarcinoma	Signet ring cell carcinoma
Observation group	53	30	23	42–68	50.11 ± 5.13	32	12	9
Control group	53	27	26	43–66	49.98 ± 5.34	34	11	8
*t*	—	0.130						
*P*	—	0.897						

**Table 2:** Comparison of effectiveness (%).

Groups	*n*	CR	PR	SD	PD	Total
Observation group	53	22 (41.51)	24 (45.28)	6 (11.32)	1 (1.89)	46 (86.79)
Control group	53	10 (18.87)	15 (28.30)	21 (39.62)	7 (13.21)	25 (47.16)
*x* ^2^	—	18.811				
*P*	—	＜0.001				

**Table 3:** Comparison of CEA and CA19-9 levels ($\bar{x}$ ± *s*).

Groups	*n*	Before treatment		After treatment	
		CEA	CA19-9	CEA	CA19-9
Observation group	53	15.23 ± 2.96	80.23 ± 9.25	2.08 ± 0.47^*∗*^	15.12 ± 6.74^*∗*^
Control group	53	15.17 ± 3.13	79.89 ± 9.47	5.46 ± 1.84^*∗*^	31.82 ± 7.48^*∗*^
*t*	—	0.085	0.187	12.975	12.068
*P*	—	0.932	0.852	＜0.001	＜0.001

Note: ^*∗*^ indicates that there is a statistically significant difference in the same group before and after treatment, *P* < 0.05.

## Data Availability

The datasets used during the present study are available from the corresponding author upon reasonable request.
